The article "Salinity-induced changes in the morphology and major mineral nutrient composition of purslane (Portulaca oleracea L.) accessions" was retracted in 2023. Reason: duplicate publication.

# Salinity-induced changes in the morphology and major mineral nutrient composition of purslane (*Portulaca oleracea* L.) accessions

**DOI:** 10.1186/s40659-016-0084-5

**Published:** 2016-04-18

**Authors:** Md. Amirul Alam, Abdul Shukor Juraimi, M. Y. Rafii, Azizah Abdul Hamid, Farzad Aslani, M. A. Hakim

**Affiliations:** School of Agriculture Science and Biotechnology, Faculty of Bioresources and Food Industry, Universiti Sultan Zainal Abidin, Tembila Campus, 22200 Besut, Terengganu Malaysia; Department of Crop Science, Faculty of Agriculture, Universiti Putra Malaysia, UPM Serdang, 43400 Serdang, Selangor, DE Malaysia; Institute of Tropical Agriculture, Universiti Putra Malaysia, UPM Serdang, 43400 Serdang, Selangor, DE Malaysia; Faculty of Food Science and Technology, Universiti Putra Malaysia, UPM Serdang, 43400 Serdang, Selangor, DE Malaysia

**Keywords:** Purslane (*Portulaca oleracea* L.), NaCl, Salinity, Morphology, Mineral compositions

## Abstract

This study was undertaken to determine the effects of varied salinity regimes on the morphological traits (plant height, number of leaves, number of flowers, fresh and dry weight) and major mineral composition of 13 selected purslane accessions. Most of the morphological traits measured were reduced at varied salinity levels (0.0, 8, 16, 24 and 32 dS m^−1^), but plant height was found to increase in Ac1 at 16 dS m^−1^ salinity, and Ac13 was the most affected accession. The highest reductions in the number of leaves and number of flowers were recorded in Ac13 at 32 dS m^−1^ salinity compared to the control. The highest fresh and dry weight reductions were noted in Ac8 and Ac6, respectively, at 32 dS m^−1^ salinity, whereas the highest increase in both fresh and dry weight was recorded in Ac9 at 24 dS m^−1^ salinity compared to the control. In contrast, at lower salinity levels, all of the measured mineral levels were found to increase and later decrease with increasing salinity, but the performance of different accessions was different depending on the salinity level. A dendrogram was also constructed by UPGMA based on the morphological traits and mineral compositions, in which the 13 accessions were grouped into 5 clusters, indicating greater diversity among them. A three-dimensional principal component analysis also confirmed the output of grouping from cluster analysis.

## Background

Purslane (*Portulaca oleracea* L.) is the eighth most common plant distributed throughout the world, because it is an important heat- and drought-tolerant vegetable crop [9]. It is eaten fresh, cooked or dried, and cultivation has gained popularity across the world in recent years because the plant has been identified as a rich source of ω3 poly-unsaturated fatty acids and antioxidants [3, 49]. Moreover, purslane is promising for providing both novel biologically active substances and essential compounds for human nutrition [15]. Purslane has proven to be more salt-tolerant than any other vegetable crop [4, 58] and can produce sufficient biomass under moderate salinity stress, which other vegetable crops cannot [32]. Salinity is possibly the most significant ecological factor that causes extensive crop yield losses globally, and its threat is escalating daily [48]. Increasing salinity reduces the average yield of major crops by more than 50 % [14], and these losses are of great concern, mainly in countries with agriculture-based economies. High concentrations of salt impose both osmotic and ionic stresses on plants, which lead to several morphological and physiological changes [30]. A clear stunting of plants has been observed to result from salinity stress [51]. Parida and Das [42] reported that the detrimental effects of high salinity in plants can result in plant death and/or decreased productivity. The earliest response is a reduction in the rate of leaf surface expansion, followed by a cessation of expansion as the stress intensifies [42]. Salinity stress causes an imbalance in the uptake of mineral nutrients and their distribution within the plants [23]. Furthermore, many nutrient interactions in salt-stressed plants can occur, which may have important consequences for growth [43]. Internal concentrations of major nutrients and their uptake have been frequently studied [17], but the relationship between micro-nutrient concentrations and soil salinity is rather complex and remains poorly understood [53]. Munns and Tester [41] stated that salt-tolerant species are able to grow and reproduce even in oceanic-level salinities. The only way to control the salinization process and to maintain the sustainability of landscapes and agricultural fields is to combat the salinization problems using environmentally safe and clean techniques and by using salt-tolerant species [13, 26]. Salt tolerant crop varieties are becoming essential in many areas of the world, including Malaysia, because of salt accumulation in soil, restrictions on groundwater use and saltwater intrusion into groundwater [29, 56]. Under the prevailing conditions of increasing salinity, it is necessary to incorporate salt-tolerant plants, which can withstand the increasing stress of salinity and can economically substitute existing crops. Therefore, this research was undertaken to study the effect of salinity on the morphological traits and mineral composition of purslane.

## Results

### Purslane morphological traits analysis

#### Plant height

The plant height of untreated control 13 purslane accessions differed very significantly (*P* < 0.0001) and ranged from 33.4 to 70 cm, with the highest plant height occurring in Ac9 and the lowest in Ac13 (Table 1). At the end of the salinity treatment, the plant height was highly reduced at 32 dS m^−1^ salinity followed by 24, 16 and 8 dS m^−1^ compared to the control plants (Table 1). However, some exceptions were also observed in the case of accession numbers Ac1, Ac2 and Ac8. Among all the 13 purslane accessions, the highest plant height reduction (>33 %) was recorded in Ac13 at 32 dS m^−1^ salinity, whereas the lowest reduction (3.28 %) was found in Ac5 at 8 dS m^−1^ salinity; both samples were ornamental purslane (Table 1). Interestingly, a slight increase (2.09 %) in plant height was also observed in Ac1 at 16 dS m^−1^ salinity stress compared to the control. Less than a 5 % reduction was observed in the case of Ac5, Ac6 and Ac9 at 8 dS m^−1^ salinity stress, while the same was observed in Ac5 at 16 dS m^−1^ salinity. Furthermore, at 24 dS m^−1^ salinity, less than a 10 % plant height reduction was recorded in Ac2 and Ac5, and even at the highest salinity stress (32 dS m^−1^), the same reduction was noted in Ac1 and Ac2 (Table 1). On average across all accessions, a total of 6.99, 10.76, 16.23 and 20.18 % reductions in plant height were recorded, respectively, at 8, 16, 24 and 32 dS m^−1^ salinity, which were statistically significant values (*P* < 0.05; Table 1).

**Table 1:** Effect of salinity on plant height of 13 purslane accessions

Purslane accessions	Plant height (cm)				
	Salinity level (dS m^−1^)				
	0	8	16	24	32
Ac1	43.10h	38.30h (11.14)	44.0e (+2.09)	36.7f (14.85)	39.7d (7.89)
Ac2	42.80h	39.20h (8.41)	37.4g (12.62)	40.5e (5.37)	39.6d (7.48)
Ac3	45.80j	42.10g (8.08)	41.7f (8.95)	40.8e (10.92)	37.7e (17.68)
Ac4	48.10e	45.50f (5.41)	42.7ef (11.23)	41.4e (13.93)	40.5d (15.8)
Ac5	42.70h	41.30g (3.28)	41.0f (3.98)	39.8e (6.79)	37.4e (12.41)
Ac6	59.61b	56.70b (4.88)	53.4b (10.42)	50.2b (15.78)	46.4b (22.16)
Ac7	56.40c	52.40d (7.09)	49.8c (11.7)	46.7c (17.19)	43.2c (23.4)
Ac8	52.90d	28.20e (8.88)	47.5c (10.21)	45.8cd (13.42)	44.1c (16.64)
Ac9	70.0a	67.40a (3.71)	63.8a (8.86)	57.6a (17.71)	53.3a (23.86)
Ac10	59.20b	54.40c (8.11)	51.8b (12.5)	44.7d (24.49)	42.8c (27.7)
Ac11	43.80gh	41.60g (5.02)	38.4g (12.33)	36.9f (15.75)	33.7f (23.06)
Ac12	45.30fg	41.42g (8.57)	36.7f (18.98)	33.4g (26.27)	32.8f (27.59)
Ac13	33.40i	29.60i (11.38)	25.7h (23.05)	24.23h (27.46)	22.1g (33.83)
Mean	49.47a	46.011b (6.99)	44.15c (10.76)	41.44d (16.23)	39.48e (20.18)

Mean values with different lower case letters in a row are significantly different at *P* < 0.05. Values in the parentheses indicate percent compared to the untreated control (0 dS m^−1^) plants

‘+’ symbol denotes increase in plant height under salinity stress compared to control

#### Number of leaves

Highly significant (*P* < 0.001) variation was observed in the number of leaves in the untreated control and 13 purslane accessions. The largest number of leaves (555) was recorded in Ac13, which was a common purslane, and the lowest (351) was found in Ac3, which was an ornamental purslane (Table 2). The number of leaves in the salt-treated purslane accessions was substantially reduced with increasing salinity levels (Table 2). The highest reduction (43.6 %) was observed in Ac13 (common purslane) at the highest 32 dS m^−1^ salinity, whereas the lowest reduction (1.74 %) was noted in Ac11 (ornamental purslane) at 8 dS m^−1^ salinity compared to the control (Table 2). At 8 dS m^−1^ of salinity reduction, the number of leaves varied from 1.74 to 17.81 %, which increased to 4.28 to 27.69 % at 16 dS m^−1^ salinity. In contrast, less than a 10 % reduction was observed in Ac10 and Ac6 at 24 and 32 dS m^−1^ salinity, respectively (Table 2). Interestingly, a consequent and significant (*P* < 0.05) increase in number of leaves was also found in Ac5 and Ac9 with increasing of salinity levels compared to the control accessions (Table 2). The mean values of all of the accessions revealed a total of 8.31, 13.73 and 20.82 % reduction and 24.77 % increase in the number of main branches, respectively, at 8, 16, 24 and 32 dS m^−1^ salinity levels, which were statistically significant increases (*P* < 0.05; Table 2).

**Table 2:** Effect of salinity on number of leaves in 13 purslane accessions

Purslane accessions	Number of leaves				
	Salinity level (dS m^−1^)				
	0	8	16	24	32
Ac1	525.30ab	431.7bc (17.81)	381.4c (27.39)	350.7b (33.24)	333.61cd (36.49)
Ac2	501.20ab	413.8cd (17.44)	362.4c (27.69)	351.8b (29.81)	333.3cd (33.49)
Ac3	350.80de	314.2ef (10.43)	260.8d (25.66)	220.37c (37.18)	241.3ef (31.21)
Ac4	489.60ab	417.5cd (14.73)	403.3bc (17.63)	349.9b (28.53)	321.7cd (34.29)
Ac5	405.80cd	417.5cd (+2.88)	411.7bc (+1.45)	420.6ab (+3.65)	428.7a (+5.64)
Ac6	456.80bc	427.7bc (6.37)	411.8bc (9.85)	409.7ab (10.31)	411.2ab (9.98)
Ac7	490.40ab	444.2bc (9.42)	413.3bc (15.72)	388.7ab (20.74)	349.7b–d (28.29)
Ac8	527.20ab	511.1a (3.05)	489.7a (7.11)	449.3a (14.78)	431.5a (18.15)
Ac9	353.60de	361.2de (+2.15)	383.7c (+8.51)	359.8b (+1.75)	380.3a–c (+7.55)
Ac10	372.60d	363.4de (2.47)	356.7c (4.28)	348.3b (6.52)	333.4cd (10.52)
Ac11	487.80ab	479.3ab (1.74)	453.3ab (7.07)	389.9ab (20.07)	288.4de (40.88)
Ac12	282.60e	273.9f (3.08)	255.7d (9.52)	201.5c (28.69)	196.4f (30.5)
Ac13	555.40a	461.5a–c (16.91)	419.13bc (24.54)	351.4b (36.73)	313.4cd (43.57)
Mean	446.08a	409.0b (8.31)	384.84c (13.73)	353.23d (20.82)	335.61e (24.77)

Mean values with different lower case letters in a row are significantly different at *P* < 0.05. Values in the parentheses indicate percent compared to the untreated control (0 dS m^−1^) plants

‘+’ symbol denotes increase in number of leaves under salinity stress compared to control

#### Flowering

The numbers of flowers in the untreated control compared to 13 purslane accessions differed very significantly (*P* < 0.0001) and ranged between 6.63 and 63.47, with the highest flower numbers occurring in Ac12, which was a common purslane, and the lowest values were in Ac8, which was an ornamental purslane (Table 3). Highly significant reductions in the number of flowers were observed at the highest, 32 dS m^−1^, salinity compared to the control as well as at other salinity levels (Table 3). The highest reduction (96.48 %) in the number of flowers was recorded in Ac13 at the highest, 32 dS m^−1^, salinity, which was a common purslane, whereas the lowest reduction in the number of flowers (3.86 %) was observed in Ac5 at the lowest, 8 dS m^−1^, salinity compared to the control, which was an ornamental purslane (Table 3). All 13 purslane accessions and 4 salinity levels (except the control) had less than a 5 % reduction in the number of flowers recorded in Ac5 and Ac7 at 8 dS m^−1^ salinity, whereas a 15–56 % reduction occurred in the number of flowers that were observed at 16 dS m^−1^ salinity. Further augmented salinity levels at 24 and 32 dS m^−1^ salinity reductions in the number of flowers varied from 31–72 to 44–97 %, respectively, compared to the control (Table 3). The mean values of all of the accessions revealed 17.74, 37.79, 51.36 and 70.78 % reductions in the number of flowers at 8, 16, 24 and 32 dS m^−1^ salinities, respectively, which were statistically significant reductions (*P* < 0.0001; Table 3).

**Table 3:** Effect of salinity on number of flowers in 13 purslane accessions

Purslane accessions	Number of flowers				
	Salinity level (dS m^−1^)				
	0	8	16	24	32
Ac1	34.65g	26.53e (23.43)	17.23g (50.27)	13.27h (61.7)	8.92h (74.26)
Ac2	46.33c	39.63bc (14.46)	27.89e (39.8)	23.22d (49.88)	11.18f (75.87)
Ac3	33.77g	30.32g (10.22)	15.39h (54.43)	17.88f (47.05)	12.38e (63.34)
Ac4	43.28e	37.13cd (14.21)	28.6e (33.92)	19.8e (54.25)	10.58g (75.56)
Ac5	38.3f	36.82cd (3.86)	31.28c (18.33)	26.37b (31.14)	21.14a (44.8)
Ac6	44.57d	39.57bc (11.21)	34.53b (22.53)	25.55c (42.67)	17.11c (61.61)
Ac7	44.37d	42.58ab (4.03)	37.39a (15.73)	33.31a (24.93)	19.41b (56.25)
Ac8	6.63k	5.13h (22.62)	3.47j (47.66)	3.08f (53.54)	2.43j (63.35)
Ac9	18.78j	15.12g (19.48)	12.39i (34.03)	11.12i (40.78)	7.44i (60.38)
Ac10	25.53h	22.13f (13.32)	17.81g (30.24)	13.24h (48.14)	7.11i (72.15)
Ac11	23.34i	21.58f (7.54)	17.69g (24.21)	11.28i (51.67)	7.23i (69.02)
Ac12	63.47a	33.53d (47.17)	29.68d (53.24)	19.42e (69.4)	13.47c (78.78)
Ac13	57.61b	45.32a (21.33)	25.61f (55.55)	16.23g (71.83)	2.03j (96.48)
Mean	36.97a	29.39b (17.74)	23.0c (37.79)	17.98d (51.36)	10.8e (70.78)

Mean values and ± SE with different lower case letters in a row are significantly different at *P* < 0.05. Values in the parentheses indicate percent compared to the untreated control (0 dS m^−1^) plants

#### Fresh weight

Highly significant (*P* < 0.0001) variation was observed in the fresh weights in the untreated control and the 13 purslane accessions. The highest fresh weight (341.03 g) was recorded in Ac8, which was an ornamental purslane, and the lowest (103.67 g) was found in Ac13, which is a common purslane (Table 4). The fresh weights of the salinity stressed purslane accessions were also significantly affected with the highest levels (378.15 g) occurring in Ac9 at 24 dS m^−1^ salinity and the lowest (86.98 g) in Ac12 at 32 dS m^−1^ salinity compared to the control (Table 4). Increases in fresh weights with increasing salinity were recorded in Ac1 at 8 dS m^−1^ salinity, in Ac9 at 16, 24 and 32 dS m^−1^ salinity and in Ac13 at 8 and 16 dS m^−1^ salinity levels compared to the control (Table 4). At 8 dS m^−1^ salinity levels, the fresh weight reductions varied between 1 and 37 %, with the lowest reduction (0.89 %) in Ac3 and the highest (36.42 %) reduction in Ac8. In contrast, 3–43, 2–48 and 4–55 % fresh weight reductions were recorded in 16, 24 and 32 dS m^−1^ salinity, respectively. On average over all of the accessions, 14.36, 18.88, 21.02 and 26.09 % reductions in fresh weight were observed at 8, 16, 24 and 32 dS m^−1^ salinity, respectively, which were statistically significant (*P* < 0.05; Table 4).

**Table 4:** Effect of salinity on fresh weight of 13 purslane accessions

Purslane accessions	Fresh weight (g)				
	Salinity level (dS m^−1^)				
	0	8	16	24	32
Ac1	225.0e	231.33b (+2.81)	203.78b (9.43)	192.49b (14.45)	187.37b (16.72)
Ac2	213.58f	203.14e (4.88)	193.58c (9.36)	188.93bc (11.54)	171.58d (19.66)
Ac3	190.5g	188.79f (0.89)	177.93d (6.59)	181.37bc (4.79)	177.68c (6.73)
Ac4	187.0g	149.16g (20.24)	112.32g (39.94)	117.3g (37.27)	106.31h (43.15)
Ac5	134.16i	121.31h (9.58)	129.48e (3.39)	131.28f (2.15)	113.58g (15.34)
Ac6	279.0c	229.0b (17.92)	174.72d (37.38)	154.68e (44.56)	159.87e (42.69)
Ac7	230.0e	223.51c (2.82)	174.97d (23.93)	168.94d (26.55)	151.6f (34.09)
Ac8	341.03a	216.82d (36.42)	197.4bc (42.11)	180.29cd (47.13)	156.61ef (54.08)
Ac9	305.17b	248.61a (18.53)	346.97a (+13.69)	378.15a (+23.91)	355.68a (+16.55)
Ac10	149.17h	114.53i (23.22)	103.43h (30.66)	98.26h (34.13)	89.30j (40.14)
Ac11	242.0d	185.0f (23.55)	174.83d (27.76)	169.56d (29.93)	161.79e (33.14)
Ac12	129.48i	112.94i (12.77)	105.14h (18.79)	93.4h (27.27)	86.98j (32.82)
Ac13	103.66j	113.52i (+9.51)	119.81f (+15.58)	101.3h (2.78)	99.11i (4.39)
Mean	209.98a	179.82b (14.36)	170.34c (18.88)	165.84d (21.02)	155.19e (26.09)

Values with different lower case letters in a row are significantly different at *P* < 0.05. Values in the parentheses indicate percent compared to the untreated control (0 dS m^−1^) plants

‘+’ symbol indicates % increase in fresh weight compared to control

#### Dry weight

The dry matter (DM) content in the untreated control plants was significantly different (*P* < 0.0001) from the 13 purslane accessions and ranged from 7.94 to 20.67 g pot^−1^, with the highest DM content occurring in Ac6 and the lowest in Ac5 (Table 5). The dry matter content was also significantly reduced by NaCl-induced salinity stress in all 13 purslane accessions, with increasing of salinity levels occurring, except in Ac1 at 8 dS m^−1^ salinity, in Ac9 at 16, 24 and 32 dS m^−1^, in Ac12 and in Ac13 at 8 dS m^−1^ salinities, where significant increases in the dry matter content were recorded (Table 5). In contrast, the highest dry matter reduction (63.47 %) was found in Ac6 at 32 dS m^−1^ salinity, and the lowest reduction (1.64 %) was noted in Ac5 at 24 dS m^−1^ salinity, whereas the highest increase (54.19 %) in dry matter content was recorded in Ac9 at 24 dS m^−1^ salinity, following the lowest increase (1.83 %) in Ac13 at 8 dS m^−1^ salinity (Table 5). The mean values of all the accessions revealed 11.24, 20.91, 23.05 and 32.88 % reductions in the dry matter content at 8, 16, 24 and 32 dS m^−1^ salinity, respectively, which were statistically significant (*P* < 0.0001; Table 5).

**Table 5:** Effect of salinity on dry weight of 13 purslane accessions

Purslane accessions	Dry weight (g)				
	Salinity level (dS m^−1^)				
	0	8	16	24	32
Ac1	16.27bc	17.13bc (+5.29)	13.1bc (13.1)	9.23e–g (9.23)	8.33ef (8.33)
Ac2	15.39bc	13.58d (11.76)	10.34d (10.34)	9.18e–g (9.18)	8.42d–f (8.42)
Ac3	23.55a	21.39a (21.39)	19.29a (19.29)	20.16b (20.16)	18.51b (18.51)
Ac4	15.55bc	13.97cd (13.97)	10.7d (10.7)	8.95e–g (8.95)	8.66d–f (8.66)
Ac5	7.94d	6.45f (6.45)	6.74f (6.74)	7.81fg (7.81)	5.39g (5.39)
Ac6	20.67ab	17.77ab (17.77)	10.02d (10.02)	14.38c (14.38)	7.55e–g (7.55)
Ac7	15.91bc	13.24d (13.24)	14.17b (14.17)	12.77cd (12.77)	12.04c (12.04)
Ac8	16.63bc	11.57de (11.57)	11.16cd (11.16)	10.92de (10.92)	9.98c–e (9.98)
Ac9	15.5bc	13.48d (13.48)	21.3a (21.3)	23.9a (23.9)	23.4a (23.4)
Ac10	10.10cd	8.60ef (8.6)	7.44ef (7.44)	7.13g (7.13)	6.89fg (6.89)
Ac11	18.84ab	14.0cd (14.0)	13.43bc (13.43)	12.47cd (12.47)	11.08cd (11.08)
Ac12	11.99cd	14.41b–d (14.41)	9.46de (9.46)	7.72fg (7.72)	6.33fg (6.33)
Ac13	12.05cd	12.27d (12.27)	11.34cd (11.34)	9.58ef (9.58)	7.93e–g (7.93)
Mean	15.41a	13.68b (11.24)	12.19c (20.91)	11.86d (23.05)	10.35e (32.88)

Mean values with different lower case letters in a row are significantly different at *P* < 0.0001. Values in the parentheses indicate percent compared to the untreated control (0 dS m^−1^) plants

‘+’ symbol indicate % increase in dry weight compared to control

### Micro and macro mineral elements

#### Phosphorus (P) content in purslane

Significant (*P* < 0.0001) variations were also observed in the P content of the untreated control and 13 purslane accessions. The phosphorus content differed from 0.25 to 0.71 %, with the highest value observed in Ac13 and the lowest in Ac4 (Table 6). Both the negative and positive effects of different salinity levels were noted in the phosphorus content in all 13 purslane accessions. In most of the accessions, the phosphorus content was found to increase at the initial (8 dS m^−1^) augmented salinity stress, with some exceptions in Ac3, Ac4 and Ac13 compared to the control (Table 6). Further salinity increases reduced the P content in all of the purslane accessions up to the highest salinity levels, whereas a complete reduction in the P content at all 4 salinity levels was noted in Ac5 and Ac7 compared to the control (Table 6). Consequent reductions in the P contents were found to increase with increasing salinity stress, and the highest reduction (69.43 %) was seen in Ac5 at the highest salinity levels at 32 dS m^−1^, whereas the highest increase (183.07 %) was noted in Ac4 at the lowest salinity levels (8 dS m^−1^) compared to the control (Table 6). On average, over all of the accessions, 13.66 % increase, 11.61, 29.51 and 38.66 % reductions in P content were recorded, respectively, at 8, 16, 24 and 32 dS m^−1^ salinities and were statistically significant (*P* < 0.05; Table 6).

**Table 6:** Effect of salinity on P content in 13 purslane accessions

Purslane accessions	P content (%, DW basis)				
	Salinity level (dS m^−1^)				
	0	8	16	24	32
Ac1	0.32i	0.43h (+36.39)	0.14k (56.33)	0.11j (63.92)	0.11j (64.87)
Ac2	0.37g	0.42i (+14.17)	0.15j (58.86)	0.11j (69.21)	0.13h (63.49)
Ac3	0.37g	0.52f (+37.97)	0.49c (+31.02)	0.35e (7.49)	0.34c (8.56)
Ac4	0.25j	0.72a (+183.07)	0.61b (+139.76)	0.38d (+47.64)	0.23g (8.66)
Ac5	0.42d	0.20k (53.32)	0.20i (53.32)	0.15h (65.64)	0.13hi (69.43)
Ac6	0.41e	0.42i (+0.97)	0.39f (8.03)	0.32f (22.63)	0.32d (22.63)
Ac7	0.34h	0.14l (58.63)	0.13k (60.42)	0.13i (62.80)	0.12ij (63.99)
Ac8	0.54c	0.66c (+22.35)	0.40e (25.88)	0.37d (30.73)	0.25f (52.70)
Ac9	0.57b	0.59d (+3.16)	0.49c (14.91)	0.46b (19.47)	0.45a (21.40)
Ac10	0.32i	0.34j (+6.25)	0.28h (14.06)	0.24g (26.25)	0.24g (26.25)
Ac11	0.39f	0.46g (+19.74)	0.35g (9.87)	0.32f (17.14)	0.29e (25.71)
Ac12	0.42de	0.57e (+38.31)	0.41d (0.96)	0.41c (1.45)	0.37b (11.08)
Ac13	0.71a	0.70b (1.27)	0.78a (+9.31)	0.49a (31.31)	0.34c (51.76)
Mean	0.42b	0.47a (+13.66)	0.37c (11.61)	0.29d (29.51)	0.26e (38.66)

Mean values with different lower case letters in a row are significantly different at *P* < 0.05. Values in the parentheses indicate percent compared to the untreated control (0 dS m^−1^) plants

‘+’ symbol indicates % increase of P content

#### Sodium (Na) content in purslane

The accession differences in sodium concentrations in purslane were highly pronounced (*P* < 0.0001), ranging from 0.26 to 0.77 % under control conditions, with the highest in Ac11 and the lowest in Ac1 (Table 7). Sodium concentrations were observed to increase progressively with increasing salinity in most of the purslane accessions, with the exception of Ac11, where a significant decrease in the Na concentration was found at all 4 salinity levels compared to the control (Table 7). In salinity-stressed purslane, the highest increase (257.6 %) in Na concentration was observed in Ac1 at 32 dS m^−1^ salinity, whereas zero effect from salinity stress was recorded in Ac6 at 24 dS m^−1^ salinity compared to the control (Table 7). On the contrary, at the beginning in Ac13, a significant increase in Na concentration was observed; however, further increased salinity resulted in Na concentrations that declined significantly compared to the control (Table 7). On average over all of the accessions, 34.8, 54.5, 56.1 and 68.5 % increases in Na concentrations were recorded, respectively, at 8, 16, 24 and 32 dS m^−1^ salinities and were statistically significant (*P* < 0.05; Table 7).

**Table 7:** Effect of salinity on Na content in 13 purslane accessions

Purslane accessions	Na content (%, DW basis)				
	Salinity level (dS m^−1^)				
	0	8	16	24	32
Ac1	0.26l	0.46i (+72.12)	0.63f (+141.22)	0.85c (+225.57)	0.94a (+257.63)
Ac2	0.46d	0.61d (+31.61)	0.72d (+54.69)	0.86b (+85.18)	0.90b (+95.33)
Ac3	0.32j	0.34k (+7.19)	0.63f (+97.50)	0.72g (+124.69)	0.79e (+146.56)
Ac4	0.29k	0.55g (+91.29)	0.50i (+73.52)	0.73f (+153.31)	0.75g (+160.63)
Ac5	0.43f	0.59e (+36.47)	0.71e (+63.28)	0.76e (+75.98)	0.71i (+63.05)
Ac6	0.43g	0.71b (67.61)	0.62g (+44.37)	0.43l (0.0)	0.71h (+67.61)
Ac7	0.62b	0.72a (+17.40)	0.76b (+24.23)	0.86a (+40.16)	0.76f (+23.41)
Ac8	0.35h	0.36j (+3.15)	0.97a (+178.80)	0.61j (+73.35)	0.67k (+41.40)
Ac9	0.32j	0.58f (+80.56)	0.72d (+124.14)	0.83d (+160.19)	0.88c (+174.95)
Ac10	0.33i	0.54h (62.19)	0.44k (+32.04)	0.65i (+95.51)	69.2d (+107.19)
Ac11	0.77a	0.71b (7.64)	0.71c (5.96)	0.20m (74.74)	0.43l (44.43)
Ac12	0.49c	0.68c (+38.89)	0.49j (0.00)	0.68h (+38.89)	0.70j (+43.0)
Ac13	0.44e	0.57f (+29.38)	0.61h (+36.97)	0.44k (1.10)	0.37m (17.73)
Mean	0.42d	0.57c (+34.75)	0.65b (+54.51)	0.66b (+56.14)	0.71a (+68.49)

Mean values with different lower case letters in each column are significantly different at *P* < 0.05. Values in the parentheses indicate percent compared to the untreated control (0 dS m^−1^) plants

‘+’ symbol indicates % increase of Na content

#### Potassium (K) content in purslane

The potassium content varied greatly (*P* < 0.0001) among all 13 untreated purslane accessions, with the highest content (8.20 %) observed in Ac11, and the lowest content (3.30 %) in Ac1. Interestingly, the K content in Ac10 (an ornamental purslane) and in Ac12 (a common purslane) was found to be similar (5.98 %), which was also statistically non-significant. Augmented salinity stresses also significantly (*P* < 0.05) reduced the K content in all 13 purslane accessions, except in Ac1 and Ac10 at 8 dS m^−1^ salinity, in which a slight increase (4.51 and 8.79 %, respectively) in the K content was recorded compared to the control (Table 8). Throughout the salinity treatments, the K contents were increasingly reduced with increasing salinity levels, and the highest reduction (60.6 %) was observed in Ac5 at 32 dS m^−1^ salinity, whereas the lowest (0.84 %) was seen in Ac12 at the lowest (8 dS m^−1^) salinity stress compared to the control (Table 8). On average, over all of the accessions, 13.08, 25.18, 31.93 and 37.40 % reductions in K content were recorded, respectively, at 8, 16, 24 and 32 dS m^−1^ salinity and were statistically significant values (*P* < 0.05; Table 8).

**Table 8:** Effect of salinity on K content in 13 purslane accessions

Purslane accessions	K content (%, DW basis)				
	Salinity level (dS m^−1^)				
	0	8	16	24	32
Ac1	3.33h	3.48f (+4.51)	3.18h (4.51)	2.80d (15.79)	2.55h (23.31)
Ac2	3.8g	3.48f (8.55)	3.13h (17.76)	2.83d (25.66)	2.65h (30.26)
Ac3	5.78de	5.35d (7.36)	4.13f (28.57)	4.03c (30.30)	3.75de (35.06)
Ac4	7.18b	5.05e (29.62)	4.70d (34.49)	4.05c (43.55)	3.40f (52.61)
Ac5	6.30c	3.70f (41.27)	3.05h (51.59)	2.90d (53.97)	2.48h (60.60)
Ac6	5.15f	4.88e (5.34)	4.48e (13.11)	4.00c (22.33)	3.10g (39.81)
Ac7	5.60e	3.78f (32.59)	3.60g (35.71)	3.20d (42.86)	2.98g (46.88)
Ac8	5.18f	5.08d (1.93)	4.95c (4.35)	4.50bc (13.04)	4.13bc (20.29)
Ac9	6.28c	5.88c (6.37)	5.40a (13.94)	5.10a (18.73)	6.50a (+3.59)
Ac10	5.98d	6.50b (+8.79)	5.15bc (13.81)	4.34bc (27.33)	4.30b (28.03)
Ac11	8.20a	7.70a (6.10)	4.98c (39.33)	4.80ab (41.46)	3.55ef (56.71)
Ac12	5.98d	5.93c (0.84)	5.23ab (12.55)	4.48bc (25.10)	4.00cd (33.05)
Ac13	7.33b	5.33d (27.30)	4.95c (32.42)	4.75ab (35.15)	4.23bc (42.32)
Mean	5.85a	5.08b (13.08)	4.38c (25.18)	3.98d (31.93)	3.66e (37.40)

Mean values with different lower case letters in a row are significantly different at *P* < 0.05. Values in the parentheses indicate percent compared to the untreated control (0 dS m^−1^) plants

‘+’ symbol indicates % increase of K content

#### Calcium (Ca) content in purslane

Calcium concentrations in purslane accessions observed in the range of 4.17–1.40 % in untreated control plants with the highest levels in Ac6 and the lowest in Ac10 (Table 9). The calcium content was heavily affected by salinity, with clear differences among accessions where both an increase and decrease in Ca concentrations were observed (Table 9). An increase in Ca concentrations throughout the 4 salinity levels was found in Ac4, Ac9, Ac10, Ac12 and Ac13. However, in Ac7, the only increase was seen at 24 dS m^−1^ salinity and in Ac8 at 8 and 16 dS m^−1^ salinity, compared to the control. However, the highest increase (145 %) in Ca concentration due to salinity stress was observed in Ac10 at 8 dS m^−1^ salinity, followed by 123 % increase in Ac13 and 109 % increase in Ac10 at 32 dS m^−1^ salinity compared to the control (Table 9). However, the highest decrease (61 %) in Ca concentration was recorded in Ac1 at 24 dS m^−1^ salinity followed by 58.8 % decrease at 16 dS m^−1^ salinity in the same accession and a 55 % decrease in Ac5 at 8 dS m^−1^ salinity compared to the control (Table 9). On average over all of the accessions, 3.73 % increase, 8.38 % decrease, 5.76 % and 2.23 % increase in Ca concentration were recorded, respectively, at 8, 16, 24 and 32 dS m^−1^ salinity, which were statistically significant values (*P* < 0.05; Table 9).

**Table 9:** Effect of salinity on Ca content in 13 purslane accessions

Purslane accessions	Ca content (%, DW basis)				
	Salinity level (dS m^−1^)				
	0	8	16	24	32
Ac1	2.74f	1.65i (39.80)	1.13k (58.77)	1.06l (61.11)	1.33l (51.46)
Ac2	1.94i	1.72i (11.33)	1.60j (17.59)	1.60k (17.59)	1.25m (35.72)
Ac3	3.28b	2.13g (34.93)	3.06b (6.83)	2.49g (24.15)	2.38g (27.32)
Ac4	2.08h	3.72b (+78.85)	2.68d (+28.85)	3.09e (+48.86)	3.17d (+52.31)
Ac5	2.72f	1.22j (55.32)	2.01h (26.22)	1.67j (38.57)	1.92j (29.45)
Ac6	4.17a	2.70e (35.12)	2.38f (42.99)	3.35c (19.58)	3.88b (6.91)
Ac7	2.66g	1.84h (30.72)	2.18g (18.07)	3.69b (+38.86)	2.12h (20.18)
Ac8	2.82e	3.62c (+28.41)	3.07b (+9.09)	2.50g (11.36)	1.65k (41.48)
Ac9	3.02d	4.20a (+39.26)	3.46a (+14.85)	5.26a (+74.27)	5.14a (+70.29)
Ac10	1.40l	3.43d (+145.14)	1.60j (+14.29)	2.36h (+68.57)	2.93e (+109.14)
Ac11	3.07c	2.55f (16.83)	1.90i (38.0)	1.93i (37.22)	1.98i (35.66)
Ac12	1.73j	3.49d (+101.85)	2.83c (+63.89)	3.22d (+86.11)	2.79f (+61.57)
Ac13	1.48k	2.06g (+38.86)	2.42e (+63.78)	2.79f (+88.65)	3.312c (+123.35)
Mean	2.55c	2.64ab (+3.73)	2.33e (8.38)	2.69a (+5.76)	2.60c (+2.23)

Mean values with different lower case letters in a row are significantly different at *P* < 0.05. Values in the parentheses indicate percent compared to the untreated control (0 dS m^−1^) plants

‘+’ symbol indicates % increase of Ca content

#### Magnesium (Mg) content in purslane

The Mg content in 13 untreated purslane accessions also significantly (*P* < 0.0001) varied, with the highest concentration (2.03 %) observed in Ac1 and the lowest concentration (0.82 %) in Ac2 (Table 10). The Mg concentration in the purslane accessions was also significantly (*P* < 0.05) affected by augmented salinity stress. The highest salinity stress increase (83 %) in Mg concentration was observed in Ac13 at 16 dS m^−1^ salinity followed by a 64.8 % increase in Ac12 at the same salinity and a 48.4 % increase in Ac13 at 24 dS m^−1^ salinity compared to the control (Table 10). In contrast, the highest reduction (61 %) in Mg content due to salinity stress was observed in Ac1 at 24 dS m^−1^ salinity followed by 60.5 % at 32 dS m^−1^ salinity and 56 % at 16 dS m^−1^ salinity in the same accessions, respectively, compared to the control (Table 10). On average, over all of the accessions, 8.92, 1.83, 5.38 and 10.35 % reductions in Mg concentration were recorded, respectively, at 8, 16, 24 and 32 dS m^−1^ salinity and were statistically significant (*P* < 0.05; Table 10).

**Table 10:** Effect of salinity on Mg content in 13 purslane accessions

Purslane accessions	Mg content (%, DW basis)				
	Salinity level (dS m^−1^)				
	0	8	16	24	32
Ac1	2.03a	1.29g (36.41)	0.89j (56.21)	0.79l (61.14)	0.80k (60.55)
Ac2	0.82k	0.93j (+13.58)	1.04h (+27.45)	1.06k (+29.90)	0.85j (+3.92)
Ac3	1.83c	1.19h (34.79)	0.90i (50.77)	1.43g (21.66)	1.56c (14.44)
Ac4	1.92b	1.89a (1.25)	1.37f (28.60)	1.69a (11.90)	1.41g (26.30)
Ac5	1.44f	1.29g (10.03)	1.36f (5.01)	1.29j (10.31)	1.15i (20.6)
Ac6	1.59d	1.36cd (14.32)	1.89a (+18.59)	1.52e (4.77)	1.61b (+1.01)
Ac7	1.38g	1.32f (4.07)	1.51c (+9.88)	1.58d (+15.12)	1.43f (+3.78)
Ac8	1.36g	1.64b (+19.94)	1.41e (+3.52)	1.32i (2.93)	1.38h (+1.47)
Ac9	1.48e	1.38c (7.01)	1.48d (0.00)	1.61c (+8.36)	1.48d (0.00)
Ac10	1.57d	1.36de (13.59)	1.51c (3.65)	1.65b (+4.95)	1.74a (+11.14)
Ac11	1.03h	1.15i (+10.93)	1.32g (+27.47)	1.40h (+35.61)	1.46e (+41.81)
Ac12	0.92j	0.58k (36.52)	1.52c (+64.78)	0.56 m (39.13)	0.80k (13.48)
Ac13	0.99i	1.34ef (34.88)	1.82b (+83.06)	1.47f (+48.39)	0.77l (221.90)
Mean	1.41a	1.29d (8.92)	1.39b (1.84)	1.34c (5.38)	1.27e (10.35)

Mean values with different lower case letters in a row are significantly different at *P* < 0.05. Values in the parentheses indicate percent compared to control (0 dS m^−1^) plants

‘+’ symbol indicates % increase of Mg content

#### Iron (Fe) content in purslane

Thirteen untreated control purslane accessions greatly varied in Fe concentration and ranged between 9.30 and 56.0 ppm, with the highest concentration observed in Ac6 and the lowest in Ac7 (Table 11). Varied levels of salinity also significantly (*P* < 0.05) affected the Fe concentration. At 8 dS m^−1^ salinity, the Fe content was found to increase in all purslane accessions, except Ac1, where a decrease in Fe content was recorded at all salinity levels. At this lower salinity level, the highest increase (344.8 %) in Fe content was seen in Ac5, followed by 278 % in Ac4, respectively, compared to the control (Table 11). However, a further increase in salinity also continued to increase the Fe content in Ac4, Ac5, Ac7, Ac8, Ac9, Ac10 and Ac13 but at a decreasing rate. However, Ac2, Ac3, Ac6, Ac11 and Ac12 exhibited reductions in Fe content when the salinity levels changed to 16  dS m^−1^ from 8 dS m^−1^ (Table 11). Furthermore, NaCl-induced the highest reduction (74.9 %) in Fe content in Ac6 at 32 dS m^−1^ salinity, followed by a 64 % reduction in Ac3 at the same salinity levels compared to the control (Table 11). On average, over all of the accessions, 66.7 and 10.5 % increases at 8 and 16 dS m^−1^ salinity, and 21 and 35.7 % reductions in Fe concentrations were recorded at 24 and 32 dS m^−1^ salinity, respectively, which were statistically significant (*P* < 0.05; Table 11).

**Table 11:** Effect of salinity on Fe content in 13 purslane accessions

Purslane accessions	Fe content (ppm)				
	Salinity level (dS m^−1^)				
	0	8	16	24	32
Ac1	25.70e	21.90i (14.79)	19.80h (22.92)	14.60g (43.19)	12.20gh (52.53)
Ac2	26.30e	42.40f (+61.22)	19.70h (25.10)	21.80cd (17.11)	29.80b (+13.31)
Ac3	28.60d	45.60e (+59.44)	19.50h (31.82)	18.30f (36.01)	10.20hi (64.34)
Ac4	16.90g	63.90b (+278.11)	28.10f (+66.27)	19.80ef (+17.16)	14.60ef (13.61)
Ac5	14.50h	64.50b (+344.83)	42.7b (+194.48)	20.9de (+44.14)	16.20de (+11.72)
Ac6	55.50a	91.40a (+64.68)	39.50c (28.83)	25.80b (53.51)	13.90fg (74.95)
Ac7	9.30i	16.70j (+79.57)	15.70j (+68.82)	11.10i (+19.35)	23.40c (+151.61)
Ac8	30.70d	33.80h (+10.10)	30.90e (+0.65)	33.80c (+10.10)	22.60d (26.38)
Ac9	21.40f	36.0g (+68.22)	23.10g (+7.94)	12.90h (39.72)	10.40hi (51.40)
Ac10	19.80f	44.0ef (+122.22)	22.70g (+14.65)	20.30de (+2.53)	16.00de (19.19)
Ac11	29.30d	45.80e (+56.31)	26.80f (8.53)	13.10gh (55.29)	8.40i (71.33)
Ac12	43.30c	52.00d (+20.09)	33.20d (25.33)	22.60c (47.81)	22.50c (48.04)
Ac13	50.30b	61.30c (+21.87)	88.90a (+76.74)	58.30a (+15.90)	38.70a (23.06)
Mean	28.60c	47.60a (+66.66)	31.60b (+10.50)	22.60cd (21.07)	18.40d (35.71)

Mean values with different lower case letters in a row are significantly different at *P* < 0.05. Values in the parentheses indicate percent compared to the untreated control (0 dS m^−1^) plants

‘+’ symbol indicates % increase of Fe content

#### Zink (Zn) content in purslane

The zinc content also varied greatly among all 13 untreated control purslane accessions, with the highest Zn content (0.74 ppm) in Ac12 and the lowest (0.31 ppm) in Ac9 (Table 12). Aggravated salinity stress caused significant changes in the Zn content among the purslane accessions. At the lowest salinity levels (8 dS m^−1^), an increase in Zn concentration was seen in all 13 purslane accessions compared to the control, with the highest increase (182.6 %) in Ac6 followed by a 48.6 % increase in Ac12 and 48.5 % increase in Ac7, respectively (Table 12). The Zn concentration continued to increase with further increases in salinity levels at 16 dS m^−1^ salinity in Ac1, Ac2, Ac3, Ac4, Ac5, Ac7, Ac11 and Ac12, but the Zn concentration decreased in percentage compared to the control (Table 12). Meanwhile, the highest reduction (56.6 %) in Zn content due to salinity stress was found in Ac13 at 32 dS m^−1^ salinity, followed by a 34.7 % reduction in Ac6 at 32 dS m^−1^ salinity and 33.3 % reduction in Ac8 at 16 dS m^−1^ salinity, respectively, compared to the control (Table 12). On average over all of the accessions, a 38.8 % increase, 8.95, 3.2 and 8.8 % reduction in the Zn concentration were recorded at 8, 16, 24 and 32 dS m^−1^ salinity levels, respectively, which were statistically significant (*P* < 0.05; Table 12).

**Table 12:** Effect of salinity on Zn content in 13 purslane accessions

Purslane accessions	Zn content (mg L^−1^)				
	Salinity level (dS m^−1^)				
	0	8	16	24	32
Ac1	0.43cd	0.51e–g (+18.60)	0.53bc (+23.26)	0.46b (+6.98)	0.4cd (6.98)
Ac2	0.41ed	0.49f–h (+19.51)	0.45cd (+9.76)	0.37cd (9.76)	0.33ef (19.51)
Ac3	0.4d–f	0.47gh (+17.51)	0.5bc (+25.0)	0.39bc (2.50)	0.46bc (+15.0)
Ac4	0.35e–g	0.62c (+77.14)	0.4d (+14.29)	0.38cd (+8.57)	0.4cd (+14.29)
Ac5	0.49bc	0.54de (+10.20)	0.56b (+14.29)	0.44bc (10.20)	0.52b (+6.12)
Ac6	0.46b–d	1.3a (+182.61)	0.46cd (0.00)	0.42bc (8.70)	0.3f (34.78)
Ac7	0.33fg	0.49f–h (+48.48)	0.48b–d (+45.45)	0.37cd (+12.12)	0.36de (+9.09)
Ac8	0.42c–e	0.52de (+23.81)	0.28e (33.33)	0.31d (26.19)	0.3f (28.57)
Ac9	0.31g	0.23i (25.81)	0.28e (9.68)	0.38cd (+22.58)	0.38de (+22.58)
Ac10	0.44cd	0.45h (+2.27)	0.41d (6.82)	0.42bc (4.55)	0.32ef (27.27)
Ac11	0.39d–f	0.56d (+43.59)	0.48b–d (+23.08)	0.37cd (5.13)	0.35de (10.26)
Ac12	0.74a	1.1b (+48.68)	0.93a (+25.68)	0.84a (+13.51)	0.85a (+14.86)
Ac13	0.53b	0.63c (+18.87)	0.45cd (15.09)	0.37cd (30.19)	0.23g (56.60)
Mean	0.44c	0.61a (+38.77)	0.48b (8.95)	0.42d (3.16)	0.40d (8.77)

Mean values with different lower case letters in a row are significantly different at *P* < 0.05. Values in the parentheses indicate percent compared to the untreated control (0 dS m^−1^) plants

‘+’ symbol indicates % increase of Zn content

#### Salt salinity relationships

The sodium–calcium ratio was found to increase with lower levels of salinity but decreased polynomially (R^2^ = 0.956) at the highest level of salinity (Fig. 1). The sodium–potassium ratio was influenced by the different levels of salinity in purslane and the ratios increased polynomially (R^2^ = 0.994) with salinity (Fig. 1). The potassium–phosphorus ratio declined with lower levels of salinity stress but later tended to increase polynomially (R^2^ = 0.854) with increased salinity levels (Fig. 1). The magnesium–calcium ratio decreased initially but later increased with increasing salinity levels (R^2^ = 0.909) (Fig. 1). The zinc to iron ratio was also found to decrease at the beginning of salinity stress but to later increase polynomially (R^2^ = 0.935) with increasing salinity levels (Fig. 1).

**Fig. 1:** Relationship between salinity and cation levels measured in purslane (pooled across accessions)

### Correlation matrix

The correlation matrixes for seven mineral cations in purslane at different salinity levels are presented in Table 13. Phosphorus had a strong positive correlation (*P* ≤ 0.001) with potassium and was negatively correlated (*P* ≤ 0.05) with sodium and positively correlated (*P* ≤ 0.05) with calcium and iron, whereas no statistically significant correlation was found with magnesium and zinc. Whereas potassium was significantly correlated (*P* ≤ 0.05) with sodium and calcium, the positive correlations observed with magnesium and iron and the negative associations observed with zinc were not statistically significant. In contrast, sodium was negatively correlated with iron (Table 13).

**Table 13:** Pearson’s correlation coefficients between micro and macro minerals

Factors	P	K	Na	Ca	Mg	Fe	Zn
P	1						
K	0.73**	1					
Na	−0.62*	−0.56*	1				
Ca	0.61*	0.64*	−0.09 ns	1			
Mg	0.14 ns	0.30 ns	−0.26 ns	0.50 ns	1		
Fe	0.58*	0.21 ns	−0.59*	0.07 ns	−0.05 ns	1	
Zn	0.04 ns	−0.03 ns	−0.09 ns	−0.02 ns	−0.50 ns	0.30 ns	1

*ns* non-significant

*, ** Significance at 5 and 1 % levels, respectively

### Cluster and principal component analysis (PCA)

To assess the patterns of variation, a UPGMA cluster analysis and PCA were performed using the measured parameters. All 13 purslane accessions were grouped into five distinct clusters at a 1.19 similarity coefficient level (Fig. 2). Among the 5 clusters, Ac9 was separated from the others and formed cluster V, Ac12 solely constituted cluster IV, and Ac13 was alone in cluster III. Cluster II was the largest group, consisting of Ac3, Ac4, Ac8, Ac10, and Ac11. The cluster I was formed with Ac1, Ac2, Ac5 and Ac7. The biplot of the 13 salinity tolerant purslane accessions, representing the variations among the measured parameters, are shown in Fig. 3. The patterns of the cluster analysis were also confirmed with a PCA with a three-dimensional (3D, Fig. 4) plot, which also gave results similar to those of the dendrogram (Fig. 2). The principal components analysis (PCA) confirmed 82.9 % of the total variation among all of the accessions studied (Table 14).

**Fig. 2:** A UPGMA dendrogram of measured traits derived from 13 salinity tolerant purslane accessions

**Fig. 3:** The biplot of the 13 salinity tolerant purslane accessions representing the variations among measured parameters

**Fig. 4:** A three-dimensional PCA plot indicating variations among 13 salinity tolerant purslane accessions

**Table 14:** Principal component analysis and percentage variation with first four principal components for 13 purslane accessions

Variable	Eigen vector			
	PC1	PC2	PC3	PC4
Eigen value	39.81	31.61	17.78	10.3
Percent	33.2	26.3	14.8	8.6
Cumulative	33.2	59.5	74.3	82.9
Ph	0.429	−0.156	0.058	−0.25
#Leaf	0.112	−0.137	−0.623	−0.153
#Flower	−0.314	−0.077	0.181	−0.632
FW	0.422	−0.164	0.134	0.086
DW	0.36	0.027	0.33	0.075
Na	0.068	−0.471	0.237	−0.161
P	0.114	0.505	0.047	0.102
K	0.196	0.439	0.057	0.103
Ca	0.34	0.275	0.247	−0.372
Mg	0.297	0.109	−0.33	−0.472
Fe	−0.208	0.386	−0.189	−0.234
Zn	−0.308	0.129	0.427	−0.195

## Discussions

Important morphological traits, i.e., plant height, number of leaves, number of flowers, fresh weight and dry weight, and concentrations of major macro- and micro-minerals, i.e., Na, P, K, Ca, Mg, Fe and Zn, in 13 untreated and salt-treated purslane accessions were investigated in this study. The results indicated that the untreated control plants greatly varied in the above-mentioned parameters representing morphological traits and mineral contents. Salt treatment also significantly influenced all of the investigated parameters in this study. The responses of the 13 purslane accessions to salt treatment were very different from each other and did not follow any particular trend, indicating vast diversity among the purslane accessions collected from different locations in western peninsular Malaysia.

Among the morphological traits, plant height varied greatly in the untreated control 13 purslane accessions. The plant heights ranged from 33 to 70 cm (an approximately twofold difference from lowest to highest, Table 1); the number of leaves ranged from 282 to 556 (an approximately twofold difference from lowest to highest, Table 2); the number of flowers ranged from 6 to 64 (an approximately tenfold difference from lowest to highest, Table 3). The fresh weight varied from 103 to 342 g (an approximately fourfold difference from lowest to highest, Table 4) and the dry weight ranged from 7 to 24 g (an approximately threefold difference from lowest to highest, Table 5).

NaCl-induced salinity had significant impacts on the plant height, number of leaves, numbers of flowers, fresh weights and dry weights of the 13 purslane accessions. However, the responses of the individual accessions were very different from each other. One general trend was that treatments with the highest 32 dS m^−1^ salinity caused significant reductions in all measured traits for most accessions compared to 24 dS m^−1^ salinity. The effects of 8, 16 and 24 dS m^−1^ salinity were variable; either increasing or declining (or remaining similar) in these parameters compared to the untreated control plants. An increase in plant height was recorded only in Ac1 at 16 dS m^−1^ salinity and was a very small increase (2 %) compared to the control. Consecutive and significant decreases in plant height were observed in the remaining 12 purslane accessions. At 8 and 16 dS m^−1^ salinity, the highest reduction (>46 and >48 %, respectively) was observed in Ac8 compared to the control and to all other accessions (Table 1). Ali et al. [7] and Kafi and Rahimi [32] reported significant plant height reductions in purslane at 24 mM of salinity stress. Salinity stress-induced reductions in plant height have also been observed in rice [24] and in turfgrass [55, 56]. In contrast, 13.17 % increases in plant height in *Pennisetum alopecuroides* grass at 100 mM salinity stress have been described by Mane et al. [34].

Purslane is a succulent, leafy vegetable plant, and it produces an abundant number of leaves. Therefore, the shedding of leaves is the first symptom of salinity stress. Throughout the experiment, the shedding of leaves was observed to increase with increasing salinity levels from 8 up to 32 dS m^−1^ salinity. The highest reduction (43.57 %; approximately threefold higher from lowest to highest) in leaves was found in Ac13 compared to the control (Table 2). At 8 and 16 dS m^−1^ salinity levels, non-significant (*P* > 0.05) differences were observed in Ac1, Ac2, Ac4 and Ac5. However, at 24 and 32 dS m^−1^ salinity levels, Ac1, Ac2 and Ac4 varied non-significantly. Similarly, at 24 and 32 dS m^−1^ salinity, Ac10, Ac11 and Ac12 also varied non-significantly (Table 3). Ahmad et al. [1] reported a reduction in the number of leaves in *Rosa hybrida* L. due to slight increases in salinity. Augmented salinity induced a reduction in the leaf numbers in Jojoba plants following the application of a higher salinity treatment (120.7 mM NaCl) in Ali et al. [8].

The numbers of flowers also significantly varied among the 13 salinity-stressed purslane accessions throughout the experimental period. Accession-wide responses to different salinity levels were also very significant. The highest level of flower reduction was 96.48 % (approximately fivefold higher from lowest to highest) in Ac13 at 32 dS m^−1^ salinity, followed by 78.78 % (approximately twofold higher from lowest to highest) in Ac12, 75.87 % (approximately fivefold higher from lowest to highest) in Ac2, 75.56 % (approximately fivefold higher from lowest to highest) in Ac4, and 74.26 % (approximately threefold higher from lowest to highest) in Ac1 at 32 dS m^−1^ salinity, compared to the control (Table 3). Both of the common purslane varieties were the most affected accessions compared to the ornamental accessions. Very highly significant reductions in the number of flowers in Cumin (*Cuminum cyminum* L.) have been reported by Hassanzadehdelouei et al., [27] at 11 dS m^−1^ salinity. In wheat (*Triticum aestivum*), high reductions in the numbers of spikelets have also been described by Ranjbar [44] at 20 dS m^−1^ salinity. The shedding or reduction of flower numbers from salt stressed plants may be due to a lack of optimum water uptake from roots. Abiotic stresses are known to affect meiosis during gamete production and male sterility appears to be more common than female gamete sterility [46].

Purslane is a succulent plant containing approximately 90 % water or more, in both the leaves and stems. Therefore, the fresh weight of purslane was comparatively higher than the dry weight. The elevated salinity stress caused a very high and significant reduction in the fresh weight of purslane and the fresh weight reduction increased with increasing salinity augmentation. In contrast, some of the accessions also achieved a significant increase in the fresh weight of purslane after salinity application. The highest reduction in fresh weight was observed in Ac8 at all 4 salinity levels of 8 dS m^−1^ (36.43 %), at 16 dS m^−1^ (42.1 %), at 24 dS m^−1^ (47.13 %) and at 32 dS m^−1^ (54.1 %), respectively, compared to the control as well as in other accessions (Table 4). Accession fresh weight at 8–32 dS m^−1^ salinity showed 42.69 and 32.82 % reductions (approximately threefold higher from lowest to highest) were found in Ac6 and Ac12, respectively, compared to the control (Table 4). In contrast, salinity induced the highest increase in the fresh weight in Ac9 (23.9 %; approximately twofold higher from lowest to highest) at 24 dS m^−1^ salinity, but with a further increase in salinity to 32 dS m^−1^, a smaller increase of 16.5 % was seen compared to the control (Table 4). Salinity-induced fresh weight reduction is a common phenomenon that occurs in most cultivated crop plants and trees. The reductions in fresh weight due to salinity stress have been investigated by several scientists in several tomato crops [37] and in *Ocimum basilicum* [36]. The increase in fresh weight in *Pennisetum alopecuroides* at 100 mM salinity has also been reported by Mane et al. [34]. In this study, a reduction in biomass accelerated with increasing salinity, which is obvious because of the disturbances in physiological and biochemical activities under saline conditions [16], which may be due to the reduction in leaf area and number of leaves [19].

Plant dry matter content is a functional parameter that is used to assess plant strategy resource acquisition and use [20]. NaCl-induced salinity significantly affected the total dry matter production in all 13 purslane accessions. The dry matter production in purslane was very low compared to the fresh weight due to very high water content in the leaves and stems. The highest significant reduction in dry matter content (63.47 %; approximately a fivefold reduction from lowest to highest) was recorded in Ac6 at 32 dS m^−1^ salinity followed by 51.52 % (approximately a fourfold reduction from lowest to highest) in the same accessions at 16 dS m^−1^ salinity, respectively, compared to the control (Table 7). In contrast, in Ac9, a successive increase in dry matter content was noted from 16 to 32 dS m^−1^ salinity, where the highest increase (54.2 %) occurred at 24 dS m^−1^ salinity; however, the increasing rate of dry matter content later decreased with increasing salinity compared to the control (Table 5). The significant decrease in dry matter content of sugar beet cultivars was described by Dadkhah and Grrifiths [18] at 350 mM salinity stress. A level of 250 mM salinity resulted in the shoot and root dry matter contents exhibiting a marked decrease in hybrid maize varieties [21]. Worldwide, several authors have published reports on dry matter reductions in different crops under salinity stressed conditions in rice [24], turfgrass (Uddinn et al. 2012; [54]) and *Solanum quitoense* Lam. [22]. However, an increase in dry matter content in *Pennisetum alopecuroides* at 100 mM salinity has also been reported by Mane et al. [34]. This induced dry matter production under salinity conditions might be due to the accumulation of inorganic ions and organic solutes for osmotic adaptation, whereas a decrease in the dry matter content at the highest salinity levels might be due to the inhibition of hydrolysis in reserved nutrients and their translocation to the growing shoots [34].

The major micro- and macro-mineral contents of 13 untreated and salt-treated purslane accessions were also determined in our study. Clear and highly significant (*P* ≤ 0.001) accession variations were observed across all measurements of Na^+^, P, K^+^, Ca^2+^, Mg^2+^, Fe and Zn content in the untreated 13 purslane accessions. Among the measured mineral contents in purslane, the potassium content was highest, followed by the sodium, magnesium, calcium, phosphorus, iron and zinc contents (Tables 6, 7, 8, 9, 10, 11, 12). Aggravated salinity stress also had a very significant impact on all of the measured micro and macro minerals of purslane. At lower salinity stress (8 dS m^−1^), a common trend was identified: the mineral contents of P, Na^+^, Fe and Zn increased compared to the control and reductions were observed of the remaining minerals (Table 6, 7, 8, 9, 10, 11, 12). However, after applying the next salinity level (16 dS m^−1^), the mineral content of the majority of the purslane accessions reduced significantly, and only a few continued to increase, but with decreasing rates. The phosphorous content increased at 8 dS m^−1^ salinity in most of the accessions, but later increasing levels of salinity tended to significantly decrease and continued to decrease up to the highest salinity levels compared to the control (Table 6). In agreement with our findings, Zuazo et al. [59] opined that the increase in phosphorus content at lower salinity (2.5 dS m^−1^) in mango stems and Hirpara et al. [28] showed a decrease in phosphorus content in *Butea monosperma* at the highest (13 dS m^−1^) salinity stress. As in P, an increasing trend was also observed in the sodium content with increasing salinity in most of the purslane accessions, although there were also reductions in some of the accessions (Table 7). Several researchers have found that salinity stress increased the Na^+^ content in *Butea monosperma* [28], *Salvadora persica* seedlings [43], *Andrographis paniculata* plants [52] and in common purslane [55]. In contrast, the K^+^ content was very significantly reduced in most of the purslane accessions at most salinity levels, with some exceptions for certain accessions and salinity levels (Table 8). Similar results have also been described by Talei et al. [52] in *Andrographis paniculata* plants and in common purslane by Uddin et al. [55]. NaCl-induced salinity stress caused both an increase and decrease in Ca^2+^ content in this study and different accessions responded differently at various levels of salinity stress (Table 9). The augmented salinity stress increases in calcium content have been reported in *Salvadora persica* seedlings [43] and in *Andrographis paniculata* [52]. However, Uddin and Juraimi [54] found a reduction in calcium content in turfgrass species. Similar trends were also observed in the case of Mg^2+^ content in 13 salinity stressed purslane accessions (Table 10). Zuazo et al. [59] described an increase in magnesium content in mango stems but a decrease in roots in different salinity regimes. Talei et al. [52] also reported increased magnesium in *Andrographis paniculate,* and Uddin and Juraimi [54] showed a decrease in turfgrass species. The iron content significantly increased at lower salinity levels but later tended to decrease with increasing salinity levels (Table 11). The increase in Fe^2+^ concentration due to lower salinity stress in mango rootstocks has been reported by Zuazo et al. [59]. Salinity stress reductions in iron contents have also been found in prose millet in *Andrographis paniculata* plants [52]. A similar trend was also found for the zinc contents at the lowest salinity levels in all purslane accessions, except Ac9, where reductions were recorded at 8 and 16 dS m^−1^ salinity but at increased salinity levels at 24 and 32 dS m^−1^, a significant but similar state of reduction was found (Table 12). Similar results have also been described by Talei et al. [52] in *Andrographis paniculata* plants.

There are three major constraints to plant growth in saline substrates: (a) a water deficit (drought stress) arising from low water potential of saline rooting media; (b) ion toxicity associated with the excessive uptake of mainly Na^+^ and Cl^−^; and (c) nutrient imbalances [35]. Salt-stressed plants mainly adopt three mechanisms to cope with the three constraints: (a) osmotic adjustment by inorganic and/or organic solutes; (b) salt inclusion/exclusion; and (c) ion discrimination [57]. From our previous findings [3–5] among the 13 accessions in our study, two accessions (Ac7 and Ac9) were found to be salt tolerant; six accessions (Ac3, Ac5, Ac6, Ac10, Ac11 and Ac12) were moderately tolerant; and the remaining five (Ac1, Ac2, Ac4, Ac8 and Ac13) accessions were identified as moderately susceptible to salinity stress on the basis of biomass production. Osmotic adjustment through increased Na influx (Table 6) and ion discrimination, Ca/Na, Na/K and Mg/Ca in particular (Fig. 1), seem to be the key factors in salt tolerance among these purslane accessions. Continued control over Na influx and osmotic adjustment through increased Na^+^ uptake are probably both important facets of the physiology of purslane plant ability to cope with a saline environment. For instance, from among the two most salt tolerant accessions, Ac7 accumulated less Na compared to Ac9 (Table 6), which indicated the enhanced ability of Ac7 to restrict the entry of Na into the shoot, which is commonly termed “salt exclusion”. However, Ac9 exhibited a better ability to adjust osmotic balance with greater inclusion of Na in the shoots, which is commonly termed “salt inclusion”. Halophytic or salt tolerant species differ from salt-sensitive ones in having restricted uptake or the ability to transport Na^+^ and Cl^−^ to the leaves despite an effective compartmentalization of these ions. This is critical for preventing the build-up of toxic ions in the cytoplasm [11, 38]. In salt excretory plants, salt is kept away from photosynthesizing or meristematic cells. In these plants, an osmotic balance is generally achieved via extensive accumulation of organic solutes and/or inorganic ions. However, in plants where salt inclusion is the prime mechanism, the accumulation of some inorganic ions (predominantly Na^+^ and Cl^−^) regulates the osmotic adjustment [31].

However, over all genotypes, salt tolerance was not correlated with shoot Na accumulation, suggesting considerable variation in the salinity tolerance among accessions and the possible existence of a range of salt tolerant mechanisms, both between and within purslane accessions [6]. Accession Ac9, in particular, maintained better vegetative growth despite accumulating higher Na. This might indicate salt tolerance in the discontinuous distribution of Na ions from leaf to leaf and cell to cell within the leaves, as has been explained by Ashraf et al. [12]. The shoot analyses reported here suggest that a nutritional disturbance of K and Ca has a role in shoot growth inhibition and may play a role in genotypic tolerance. This study indicated that the more tolerant accessions (Ac9) had higher K and Ca accumulation (though Ac7 only had greater Ca) in saline control conditions. Jones and Gorham [31] also reported that plants with greater salt tolerance were more efficient users of K and Ca under saline conditions.

Increased Na/Ca, Na/K and Mg/Ca ratios with increasing salinity (Fig. 1) indicated ion discrimination between Na, K, Ca and Mg. This suggested that Na, K, Ca and Mg also played a role in salt tolerance in purslane. Munns and James [39] claimed that all plants discriminate to some extent between Na and K. It is therefore possible that K/Na and Ca/Na discrimination is associated with salt tolerance. Ion imbalance, particularly when caused by Ca^2+^ and K^+^, is the most important and widely studied phenomenon affected by salt stress, which is directly influenced by the uptake of Na^+^ and Cl^−^ ions [38, 40]. Ashraf et al. [12] reported that one of the most important physiological mechanisms of salt tolerance is the selective absorption of K^+^ by plants from the saline media and that the maintenance of better concentrations of K^+^ and Ca^+^ and limit on the Na^+^ uptake are vital for salt stress tolerance in plants, as has been seen in this study with purslane. Higher K^+^/Na^+^ or Ca^2+^/Na^+^ ratios are characteristic tissue salt tolerance traits and are often used as criteria for screening for salt tolerance [11, 39, 50].

Cluster analysis and PCA, as a multivariate technique, can group individuals or objects on the basis of their characteristics. Individuals with similar descriptions are mathematically congregated within the same cluster [2]. Distance, similarity and relatedness of varieties are the foundation of this method. The UPGMA constructed dendrogram revealed 5 clusters where Ac9, Ac12 and Ac13 were most different from all of the others, indicating the highest salt tolerance and the highest diversity compared to other accessions. To improve variety development, the most judicious combination can be made with Ac9, Ac12 and Ac13 with Ac1, Ac2 or Ac4 or Ac10 or Ac8 or Ac11, which would bring about the greater genetic diversity [10]. Whereas according to biplot analysis of all the measured parameters, number of leaves showed the highest correlation with fresh weight (FW) and positioned at the opposite direction of average line of the component 1 (Fig. 3). Among measured minerals K and Ca also showed highest correlation and positioned at the lower level of both component 1 and 2 (Fig. 3).

## Conclusions

In conclusion, although there were significant variations among all 13 purslane accessions among the measured parameters, in general, this research indicated high salt tolerant crop plants that are capable of producing a satisfactory amount of dry matter content, which is a fundamental requirement of any salt tolerant plant species. Throughout the experiment, accession wise complex results were found among morphological traits. Different accessions exhibited different performances under exposure to different levels of salinity stress. However, one common trend was that all of the accessions were affected at the highest salinity level compared to the control, while some were also affected at moderate or lower salinity levels. Most of the measured morphological traits were reduced under varied salinity regimes, but plant height was found to increase in Ac1 at 16 dS m^−1^ salinity and Ac13 was the most affected accession. However, the highest reduction in the leaves and number of flowers was recorded in Ac13 at 32 dS m^−1^ salinity compared to the control. The highest fresh and dry weight reductions were noted in Ac8 and Ac6 at 32 dS m^−1^ salinity, respectively, whereas the highest increase in both fresh and dry weight was found in Ac9 at 24 dS m^−1^ salinity compared to the control. In contrast, at the lower salinity levels, all of the measured minerals were found to increase and later decrease with increasing salinity, but the performances of the accessions were different with regard to the salinity levels. Overall, among all 13 purslane accessions, considering morphological development and mineral contents, Ac9 was the most salt tolerant purslane accession that produced the highest amount of fresh and dry weight, and Ac13 was the most affected accession. It was also found that ornamental purslane showed more salt tolerance than common purslane. Therefore, we can suggest both types of purslane for consumer and commercial production as a fresh vegetable source in any type of soil, especially for saline agriculture.

## Methods

### Purslane accessions and study location

There are approximately 7 types of purslane available in Malaysia. In our study, 13 different purslane accessions were collected from varied locations in western peninsular Malaysia [3]. Among those, 11 were ornamental purslane (Ac1–Ac11) and two were common purslane (Ac12 and Ac13). The experiment was conducted in a Field-2 glasshouse at the Faculty of Agriculture, at the University of Putra Malaysia (UPM) from July to October, 2013, and all of the chemical analyses were performed at the Plant Physiology and Analytic Lab, at the Department of Crop Science, in the Faculty of Agriculture, UPM, Malaysia, and the histological study was performed at the Botany Laboratory in the same department.

### Planting and cultural practices

 Seedlings of the two common purslane varieties and cuttings of the 11 ornamental purslane accessions (ornamental purslane do not produce seeds) were first grown in plastic trays filled with rice field top soils (38.96 % sand, 11.05 % silt and 49.88 % clay) with pH 4.8, 2.64 % organic carbon, 1.25 g cc^−1^ bulk density and CEC of 7.06 meq 100 g^−1^ soil. The soil nutrient status was 0.17 % total N, 5.67 ppm available P, 15.6 ppm available K, 3357 ppm Ca and 319 ppm Mg. Soil water retention was 30.72 % (wet basis) and 46.17 % (dry basis) at field capacity. The soil belonged to the Serdang series.

Five 10-day-old seedlings or cuttings for each accession were transplanted into plastic pots (24 × 22 × 20 cm) filled with the same prepared soil mentioned above. The plants were allowed to recover from transplanting shock, and full establishment occurred over 29 days. During this time, the plants were irrigated with tap water as and when necessary. No fertilizer was used. Five levels of salinity (0, 8.0, 16.0, 24.0 and 32.0 dS m^−1^) were used in this study, which were prepared using NaCl (Merck, Darmstadt, Germany) and distilled water. Salt treatment was initiated 30 days after transplanting (DAT) and continued until the end of the study. In each pot, 200 mL of saline water was applied on alternate days in the treatment. The control plants received 200 mL of distilled water. The experiment was organized in a two factorial (purslane accessions × salinity) randomized complete block designs with three replications. Whole plants were harvested from ground level, 60 days after transplanting. The plants were washed under tap water and kept in a cool dry place for 3 days and the fresh weights were recorded. After that, the samples were transferred into an oven and left for 3 days at 40 °C to avoid sudden heat burning. Finally, the oven temperature was balanced at 50 °C and left for complete drying. The dry weights of the whole plants in each treatment and replication were recorded before grinding.

### Data collection and analysis

#### Morphological data collection

##### Plant height

The average plant heights of the five plants in each pot were measured in cm from salt treated and untreated control plants. The percentages of increase and/or decrease in plant height due to salinity stress were calculated using the following formula:

$${\text{Percentage}}\;{\text{of}}\;{\text{plant}}\;{\text{height}}\;{\text{changes}}\;{ = }\;\frac{{{\text{Control}}\;{\text{treatment}}\;{\text{value}} - \;{\text{Salinized}}\;{\text{treatment}}\;{\text{value}}}}{{{\text{Control}}\;{\text{treatment}}\;{\text{value}}}} \times 100$$

##### Number of leaves

The shedding of leaves is a prominent symptom of salinity stress in purslane. The percentage of shedding of leaves compared to untreated control plants were calculated using following formula:

$${\text{Percentage}}\;{\text{of}}\;{\text{sheeding}}\;{\text{of}}\;{\text{leaves}}\;{ = }\;\frac{{{\text{Control}}\;{\text{treatment}}\;{\text{value}} - \;{\text{Salinized}}\;{\text{treatment}}\;{\text{value}}}}{{{\text{Control}}\;{\text{treatment}}\;{\text{value}}}} \times 100$$

##### Number of flowers

Purslane blooms daily, so the total numbers of flowers were counted every day and were recorded. The percentages of flower reductions were calculated using the following formula:

$${\text{Percentage of flower reduction}} = \frac{{{\text{Control treamtnet value}} - {\text{Salinized treatment value}}}}{\text{Control treatment value}} \times 100$$

##### Fresh weight

The 60-day-old harvested fresh and surface moisture-free purslane plants were weighed using an electric balance, and the mean fresh weight (FW) was calculated. The reduction in fresh biomass with the reduction percentage from salinity stress was also measured using the above formula.

##### Dry weight

The mean dry weights (DW) were calculated from the oven-dried samples. The dry matter reduction with the percentages due to salinity stress over the control was measured using the following formula:

$${\text{Percentage of dry matter reduction}} = \frac{{{\text{Control treamtnet value}} - {\text{Salinized treatment value}}}}{\text{Control treatment value}} \times 100$$

### Micro- and macro-mineral analysis

The P, Na, K, Ca, Mg, Fe and Zn contents from the control and the salinity-stressed purslane dry samples were analysed using the digestion method [33] and were determined using an Atomic Absorption Spectrophotometer (AAS; Perkin Elmer, 5100, USA). For this purpose, the ground powder samples of 0.25 g were weighed and poured into a digestion tube. Then, 5 mL of concentrated sulphuric acid (H_2_SO_4_) were added and kept overnight or at least for 2 h until the plant materials properly moistened. Then, 2 mL of 50 % hydrogen peroxide (H_2_O_2_) was slowly added and the digestion tube was placed in a digestion block, where the digester block was set to heat for 45 min at 285 °C temperature. After 45 min, the tube was removed and allowed to cool before 2 mL of 50 % H_2_O_2_ was added again. After that, it was maintained for the heating as well as cooling process and repeated until the digested solution became colourless or clear. The cleared cool sample was then filtered and the final volume was made into 100 mL by adding distilled water for the analysis.

### Multivariate analysis

A cluster analysis was performed to construct a dendrogram based on the similarity matrix data using the unweighted pair group method with arithmetic averages (UPGMA) and the *SHAN* clustering program. All of the analyses were performed with the *NTSYS*-*pc 2.10* software [45]. The binary data were also subjected to a PCA (Principal Component Analysis) to investigate the structure of our collection. The PCA of the 13 purslane accessions were calculated using the EIGEN module of *NTSYS*-*pc 2.10* software [45]. The biplot analysis was done using Past: Palaeontological Statistics software package [25].

### Statistical analysis

All recorded data were subjected to analysis of variance using the SAS statistical software package version 9.3 [47]. Data were submitted to analysis of variance (ANOVA) and the means compared by Tukey’s multiple range test (*P* < 0.05). Pearson’s correlation coefficient analyses were done to assess the associations between different parameters.

## Abbreviations

P: phosphorus
K: potassium
Ca: calcium
Mg: magnesium
Fe: iron
Zn: zinc
dS m^−1^: deci Siemens per meter
Ac: accession
NaCl: sodium chloride
UPM: Universiti Putra Malaysia
cm: centimeter
g and g cc^−1^: gram, grams per cubic centimeter
CEC: cation exchange capacity
ppm: parts per million
meq: mill equivalents
g and g^−1^: gram and per gram
Mg: milligram
DAT: days after transplanting
mL: milliliter
FW and DW: fresh weight and dry weight
AAS: atomic absorption spectrophotometer
H_2_SO_4_ and H_2_O_2_: sulfuric acid and hydrogen peroxide
SAS: statistical analysis system
ANOVA: analysis of variance
